RETRACTED

# Esoteric Connective Tissue Therapy for chronic low back pain to reduce pain, and improve functionality and general well-being compared with physiotherapy: study protocol for a randomised controlled trial

**DOI:** 10.1186/s13063-017-2055-8

**Published:** 2017-07-17

**Authors:** Christoph Schnelle, Steffen Messerschmidt, Eunice J. Minford, Kate Greenaway-Twist, Maxine Szramka, Marianna Masiorski, Michelle Sheldrake, Mark Jones

**Affiliations:** 1 School of Public Health, University of Queensland, Herston Road, Herston, QLD Australia; 2 Department of Surgery, Antrim Area Hospital, 45 Bush Rd, Antrim, BT41 2RL UK; 3 Queen’s University Belfast, University Rd, Belfast, BT7 1NN UK; 4 The Rheumatology Centre, Sydney and Nowra, Australia; 5 University of New South Wales, High Street, Kensington, NSW Australia; 6 Total Health From Inside Out Pty Ltd, Brisbane and Gold Coast, Australia; 7 Independent physiotherapist, practising in Goonellabah, Australia; 8 Independent psychologist, practising in Sunshine Coast, Australia

**Keywords:** Chronic low back pain, Low back pain, Connective tissue, Esoteric Connective Tissue Therapy, Physiotherapy, Randomised controlled trial

## Abstract

**Background:**

Low back pain causes more global disability than any other condition. Once the acute pain becomes chronic, about two-thirds of sufferers will not fully recover after 1–2 years. There is a paucity of effective treatments for non-specific, chronic low back pain.

It has been noted that low back pain is associated with changes in the connective tissue in the affected area, and a very low-impact treatment, Esoteric Connective Tissue Therapy (ECTT), has been developed to restore flexibility in connective tissue. ECTT uses patterns of very small, circular movements, to the legs, arms, spine, sacrum and head, which anecdotally are effective in pain relief. In an unpublished single-arm phase I/II trial with chronic pain patients, ECTT showed a 56% reduction in pain after five treatments and 45% and 54% improvements at 6 months and 7–9 years of follow-up respectively.

**Methods:**

The aim of this randomised controlled trial is to compare ECTT with physiotherapy for reducing pain and improving physical function and physical and mental well-being in patients with chronic low back pain.

The trial will be held at two hospitals in Vietnam. One hundred participants with chronic low back pain greater than or equal to 40/100 on the visual analogue scale will be recruited and randomised to either ECTT or physiotherapy. Four weekly treatments will be provided by two experienced ECTT practitioners (Treatment Group, 40 minutes each) and hospital-employed physiotherapy nurses (Control Group, 50 minutes).

RETRACTED

The primary outcomes will be changes in pain, physical function per the Quebec Pain Functionality Questionnaire and physical and mental well-being recorded by the Short Form Health Survey (SF-36), with mixed modelling used as the primary statistical tool because the data are longitudinal. Initial follow-up will be at either 4 or 8 months, with a second follow-up after 12 months.

**Discussion:**

The trial design has important strengths, because it is to be conducted in hospitals under medical supervision, because ECTT is to be compared with a standard therapy and because the assessor and analyst are to be blinded. The findings from this trial will provide evidence of the efficacy of ECTT for chronic low back pain compared with standard physiotherapy treatment.

**Trial registration:**

Australian New Zealand Clinical Trials Registry, ACTRN12616001196437. Registered on 30 August 2016.

**Electronic supplementary material:**

The online version of this article (doi:10.1186/s13063-017-2055-8) contains supplementary material, which is available to authorized users.

## Background

Of the 291 conditions studied in the Global Burden of Disease 2010 Study, low back pain (LBP) rates highest in terms of years lost to disability (YLD) and sixth in terms of overall burden. Because LBP has no mortality, YLD are the same as disability adjusted life years (DALYs). With a 9.4% global prevalence (95% CI 9.0–9.8), LBP causes more global disability than any other condition.

LBP has high disability weights (DW), which means that severe acute LBP is considered as disabling as non-metastatic cancer or long-term stroke consequences (DW 0.27, 0.32 with leg pain). The disability impact of severe, chronic LBP (CLBP) has been compared with amputation of both arms without treatment or with cocaine dependency (DW 0.37 with or without leg pain) [1].

CLBP arising from ergonomic exposures at work has been associated with an estimated 21.7 million DALYs in 2010 worldwide [2]. The prevalence in urban Vietnam of LBP for those aged 16 years or older was 11.2% in a WHO-ILAR study [3].

Two surveys of 4000+ households in North Carolina, USA found that the prevalence of chronic, impairing LBP rose significantly over a 14-year interval, from 3.9% in 1992 to 10.2% in 2006 [4]. Another survey showed that over 10% of Australian adults had been significantly disabled by LBP in the past 6 months [5].

### Costs

In Australia in 2008–2009, $1.2 billion, or 1.8% of selected disease-allocated health care expenditure, was attributed to back problems [6]. Contrary to clinical guidelines, many patients with LBP start incurring significant resource use and associated expenses soon after the index diagnosis [7]. In the UK, the direct health care cost of back pain in 1998 was estimated at £1632 million while informal care and of lost productivity add up to £10,668 million annually [8].

RETRACTED

### Prognosis

For a proportion of back pain patients the prognosis can be bleak. Once you take time off work for back pain you have with different medical and benefit systems a 1–10% risk of not returning to work for at least a year. Not working for 4–6 weeks leads to a 20% probability of long-term disability and not working for 6 months reduces the possibility of returning to previous work to 50%. Once the patient loses their job or has been off work for 1–2 years, a return to work is unlikely [9].

Almost two-thirds of newly identified CLBP patients do not recover within 12 months [10, 11]. For those with longer term pain, the figure has been reported at 80% [12] including mixed primary care populations [13], with 60–80% of those who consult health care providers still reporting pain 12 months later [14–16].

Cognitive factors appear instrumental in return to work rates for workers with subacute LBP; additionally, and perhaps paradoxically, going to physiotherapy has been found to reduce the chances of returning to work [17].

### Treatments

Forty-eight systematic reviews, meta-analyses and guidelines [18–66] on non-pharmacological CLBP treatments, plus a special issue of *Spine Journal* [67], revealed no treatment that consistently provides superior results for the treatment of CLBP. Overall positive recommendations exist for exercise therapy, massage, various forms of physiotherapy, cognitive behavioural therapy and, in particular, a multi-disciplinary approach. The standard treatment, physiotherapy, tends to be no better or worse than many other treatments. Therefore, there is no gold standard treatment for CLBP, and the search for an effective treatment continues. This is shown in the recently (November 2016) updated UK NICE clinical guidelines [65] for chronic LBP, summarised in the *BMJ* [68]. No treatment is recommended for CLBP, except for radiofrequency denervation under limited circumstances.

### The present study

This randomised controlled trial with treatment and control groups treated in parallel has undergone a full ethical review by the University of Queensland’s contractor, Bellberry Pty Ltd (HREC approval number EC00444).

Many scientific articles have made urgent pleas for further investigations, especially randomised controlled trials, of treatments for CLBP [1, 9, 18, 24, 69, 70].

To quote the most downloaded paper in the history of *PLoS Med* [71], “[M]ost new discoveries will continue to stem from hypothesis-generating research with low or very low pre-study odds.” Hence, it may be worthwhile to investigate new treatments that are currently not given by registered medical professionals.

RETRACTED

Such treatments are usually referred to as complementary and alternative medicine (CAM), an ill-defined group of treatments [72–74] with the difference between “complementary” and “alternative” rarely, if ever, defined. For the purposes of this article, complementary treatments are defined as working in conjunction with and in support of medical professionals, and patients are not expected to reduce their frequency of medical doctor visits; in contrast, alternative treatments aim, at least in part, to replace the work of registered medical professionals.

One approach may be to target the connective tissue (including fascia) because this represents a substantial part of the body [75] and is important in enabling physical motion [76, 77] and considered to be involved in back pain [9, p. 159, 164–6, 171–2], with fascia having rich innervation, nocireceptors and being involved in load transfer [9, p. 155, 164–5, 198]. Therefore, finding a way to treat the connective tissue may influence acute and perhaps even chronic back pain. The authors are unaware of any current treatment for LBP that specifically targets the connective tissue.

A new complementary-to-medicine technique that concentrates on treating the connective tissue was developed by Serge Benhayon in 1999 and currently has about 30 practitioners. This technique is called Esoteric Connective Tissue Therapy (ECTT) and is a gentle, hands-on treatment that claims to work by allowing connective tissue in the body to soften and return to its fluid and flexible state, which in turn decreases the compression effects on the body from tight, hard and scarred areas of injured and diseased connective tissue, thereby possibly enabling the affected body parts to resume normal, pain-free movement.

### ECTT description

Descriptions of ECTT and anecdotal references are available [78–82]. The treatment consists of small circular motions, primarily with a diameter of 2–3.5 cm, to the legs, arms and head, with the motions to the head being even smaller. Further actions involve techniques for gently holding the hip, knee, ankle, back and spine, allowing the body to adjust (align). There is some evidence that connective tissue undergoes changes in patients with CLBP [83]; hence, there is a possible mechanism to explain the effects of treatment of the connective tissue on non-specific CLBP.

ECTT and other modalities, such as Esoteric Chakra-puncture, Esoteric Massage, Esoteric Healing and the women-practitioners-only Esoteric Breast Massage, are all derived from the same underlying understanding that energy, a word which here includes consciousness, has a strong influence on humans. This is considered a truism in many alternative treatments [84], but clearly there is no scientific consensus or even much, if any, scientific evidence that there are other influences on well-being in addition to the physical and the psychological.

RETRACTED

However, theoretically speaking, if there are such influences, and if providers were to cultivate awareness and understanding of these influences, it should be possible to design treatment modalities that work substantially better than existing modalities by addressing these important and heretofore unexamined influences as a complement to the exemplary work that is done by conventional medicine.

In the experience of its practitioners, ECTT works best when done in conjunction with the patient consulting their GP and medical specialists for any diagnostic, pharmacological or surgical interventions that could be necessary, because ECTT is not a substitute for any of these interventions but a complementary intervention.

One corollary of taking into account what ECTT practitioners refer to as energy is that ECTT practitioners consider the well-being of the practitioner to be of high importance. As a result, practitioners are required to abide by a stringent code of ethics and conduct [85] that includes the following:

“… [D]uring the life of the student/practitioner as a practising individual he and she will abstain unequivocally from pornography, the use of alcohol, recreational or illicit drugs (including all forms of cannabis, ayahuasca and or alike [sic]), nicotine (cigarettes, cigars, pipe or alike) and/or any other substance that will obscure and/or alter in any way their conscious presence and centredness.”

Although the code is unorthodox in the categorical and specific nature of its prescriptive rules, similarities exist in mainstream medicine, for example in the CatholicCare Sydney code of conduct [86].

From 2006 to 2009, KG-T, a registered physiotherapist who is also ECTT-qualified, conducted an unpublished non-comparative, single-arm phase I/II study of the effect of ECTT for chronic pain, with participants receiving an ECTT session once a week for 6 weeks. After five sessions, 45 out of 51 participants reported improved pain levels on the 100-mm Visual Analogue Pain Scale (VAS) [87–89] for pain; three participants had no change and three participants deteriorated. The average pain level moved from 40.2 mm to 17.7 mm after five treatments; after 6 months to 22.2 mm and after 7–9 years in 2016 to 18.6 mm (standard deviations from 16.8 to 21.6 mm).

This 2006–2009 ECTT study by KG-T received Southern Cross University ethical approval as a long-term follow-up study (Approval Number ECN-16-026).

RETRACTED

The biggest improvement in the previous ECTT trial was from a VAS score of 80 mm to 0 mm. The worst performances were two increases in pain scores – from a score of 30 mm to 50 mm and from a score of 50 mm to 70 mm. The improvements in this study could be due to many influences, including the placebo effect, regression to the mean or other reasons. However, the result, if it turns out to be representative, would be among the more promising outcomes available, especially in light of the low-intensity nature of the intervention.

Because the previous study is a single-arm phase I/II study evaluating safety and efficacy, the next step is to perform a randomised controlled phase III study comparing ECTT with standard therapy.

SM and another practitioner of ECTT with 8 years of experience each in ECTT have been voluntarily offering ECTT treatments at two hospitals (Pacific Hospital, Hoi An and Pacific Hospital, Tam Ky) in central Vietnam, near Da Nang, over the last 4 years, and the administrator of both hospitals has indicated his willingness to provide the facilities and resources for a randomised controlled trial comparing ECTT with the standard physiotherapeutic hospital treatment of CLBP.

### Primary objective

The primary objective of the study is to compare the results of a group of participants receiving four sessions of ECTT with the results of another group of participants receiving four sessions of conventional physiotherapy treatment, with one session given each week, to determine whether ECTT results in greater improvements in pain reduction compared with the control treatment.

### Secondary objectives

Secondary objectives of the study are to compare four sessions of ECTT with four sessions of conventional physiotherapy treatment to determine whether ECTT results in larger improvements in physical and mental health as measured by the Short Form Health Survey (SF-36, a general well-being questionnaire), and in pain functionality as measured by the Quebec Back Pain Disability Scale, compared with the control treatment.

A further secondary objective of the study is to see whether any treatment effect differs between patients with initial moderate and high pain levels.

## Methods

### Trial design

This is a randomised controlled trial of four weekly sessions of ECTT with follow-up after either 4 or 8 months and a second follow-up after 12 months. Measurements will be taken at baseline, before each session and at the final follow-up. The measurements will be made by staff at the hospital who are blind to the treatment and group assignment, and not by the practitioners or researchers.

RETRACTED

The protocol conforms to Principles 1–8 of the NIH Task Force on research standards for CLBP [90] and the Australian NHMRC “National Statement on Ethical Conduct in Human Research 2007 (Updated May 2015)” [91].

A brief Standard Protocol Items: Recommendations for Interventional Trials (SPIRIT) flow diagram is provided in Fig. 1, and a populated SPIRIT checklist is provided in Additional file 1.

**Fig. 1:** SPIRIT flow diagram of the Esoteric Connective Tissue Therapy for chronic low back pain study

### Measurements

The scales to be administered are the VAS, the Quebec Back Pain Disability Scale and the two main scales of the SF-36, the Physical Component Summary and Mental Component Summary.

The Quebec Back Pain Disability Scale [92, 93] (hereafter Quebec scale) is a 0–100 scale asking 20 questions and measures functional disability “in terms of perceived difficulty associated with simple physical activities” [93].

The 0–100-mm VAS is anchored at 0 and 100, where 0 signifies no pain and 100 agonizing pain. One study [94] has argued that the minimum clinically significant difference (“a little better”, “a little worse”) is 12 mm; another has used 18 mm [95]. A third study [96] used a literature review, an expert panel and a workshop to come to the conclusion that the “minimal important change” for VAS is 15 mm and for the Quebec scale is 20 points, while a 30% improvement on either scale was considered “clinically meaningful”. Because this latter study has been the most thorough evaluation, we will adopt their definitions of minimally clinical importance and clinically meaningful change.

The SF-36 [97] has eight scales. For three of these scales, the following minimum clinically important improvements were calculated: Physical Component Scale, 2.0; Bodily Pain, 7.8; and Physical Function, 3.3 [98]. This trial adopts these values as minimum clinically important improvements.

### Intervention

#### Esoteric Connective Tissue Therapy

The treatment consists of small circular motions, primarily with a diameter of 2–3.5 cm, to the legs, arms and head, with the motions to the head being even smaller. Further actions involve techniques for gently holding the hip, knee, ankle, back and spine, allowing the body to adjust (align).

### Participants

The study population will be individuals who present during the trial period to a participating hospital as outpatients, who are over 18 years old, are not pregnant, are healthy enough to receive standard physiotherapy treatment, consent to be part of this trial and do not meet the exclusion criteria. The participants will not be charged for the treatments. The physical requirements for ECTT are lower than those for standard physiotherapy treatment; therefore, any patient who is capable of receiving the standard physiotherapy treatment is also eligible to receive ECTT. For consistency, the physical requirements are the same for both groups.

RETRACTED

#### Inclusion criteria

i. Aged 18 years or older, able to speak, read and write in Vietnamese.
ii. Suffering from CLBP, which, according to the NIH Task Force’s definition [90] is pain for at least half of the days in the past 6 months.
iii. At evaluation time, suffering from LBP at a minimum of an average of 40 out of 100 on the VAS for the previous 7 days because memory issues may appear for longer recall periods.
iv. Physically able to undertake the standard physiotherapy treatment given by the hospitals.
v. Able to complete the SF-36 questionnaire, either independently or with help from the hospital staff.

#### Exclusion criteria

i. Being pregnant or uncertain of pregnancy status.
ii. Having a clinical diagnosis of schizophrenia, bipolar conditions and/or states including mania, delirium, psychosis or any signs of psychosis, borderline disorder or major depressive disorder.
iii. Diagnosed or suspected neoplasm.
iv. Past surgery to the spine.
v. Osteoporotic fracture, neoplasm or infection, which applies to approximately 5–15% of CLBP instances [99].

#### Withdrawal criteria

Patients who withdraw after the end of week 2 will not be replaced, because the replacement would be unable to participate in four sessions. Patients who withdraw will receive normal hospital care as determined by their physician.

#### Discontinuation criteria for individuals

i. Becoming pregnant.
ii. Becoming too ill to continue.
iii. Electing not to continue.

#### Discontinuation criteria for parts of the trial or the entire trial

The trial will be stopped if a serious adverse event occurs, where ECTT is deemed to be responsible for the adverse event or where the preponderance of the evidence points to ECTT being the source.

To quote the Australian National Statement on Ethical Conduct in Human Research [91], “Serious Adverse Events” are defined as untoward medical occurrences that result in death, are life-threatening at the time, require inpatient hospitalisation or prolonging of existing hospitalisation, result in persistent or significant disability/incapacity or are medically important events or reactions.

#### Adverse events

Adverse events are recorded as part of the data collection for each session and will be reported to the clinical authorities and to the ethics committee. Participants suffering adverse events will receive free hospital care to treat the adverse event.

RETRACTED

#### Trial modifications

Important protocol modifications (e.g., changes to eligibility criteria, outcomes, analyses) will be reported to the relevant parties (investigators, trial participants, trial registry, ethics committee, journal) either immediately (investigators, trial participants) or at the time a report is due (trial registry, ethics committee, journal).

#### Data collection

The data will be entered twice by data entry personnel without identifying which are Treatment Group data and which are Control Group data and will then be compared and corrected. The statistician will then perform a number of logical and range checks and will send queries to the data entry personnel.

#### Subject confidentiality

All data will be recorded on paper and only one document will contain both the patient ID and the name and address of the patient. This document will be held by the hospital. All data entered into a computer will be in de-identified form and the data will be stored in a password-protected Microsoft Excel file and a password-protected pdf file. The statistician and any subsequent data analyst will only have access to the de-identified data.

The electronic de-identified data will be held indefinitely by the researchers for future meta-analysis and will be made accessible on a case-by-case basis with full or reduced demographic and diagnosis data depending on the circumstances

The collated data will be stored in de-identified form following the Stanford University Guidelines for electronic data collection and storage (https://web.archive.org/web/20151108213801/https://iriss.stanford.edu/onlinedataguidelines).

### Procedure

The study is a two-group, stratified, randomised, controlled study with at least 50 individuals each in a Treatment Group and a Control Group.

Patients who visit the hospital for treatment will be evaluated for their suitability for the trial and, if they are suitable and agree to participate, they will be assigned randomly to the Treatment Group or the Control Group.

The Treatment Group will receive ECTT sessions, and the Control Group will receive the conventional doctor-directed treatment, which in this design is the standard physiotherapy administered by hospital-employed physiotherapeutic nurses. The trial will use two practitioners for the ECTT Treatment Group only, because it is possible for a practitioner to treat 10 patients a day for 40 minutes each.

The stratification will be by pain level according to the VAS, with one stratum for moderate levels (40–59 mm) and another for high levels (60+ mm).

### Randomisation

For allocation, the researchers will use the website “Sealed Envelope” [100] with a block randomisation design (block size 4, 6 or 8) for 160 subjects and an overall soft limit of 100 participants. The seed used for the randomisation will be 8. The allocations will be put in 200 envelopes, which is a sufficient number in the unlikely event that an overwhelming proportion of participants are from one pain strata only. The envelopes will be marked with their pain-level stratum (moderate or high) and sequence number. The envelope will contain the group designation, with group A being the ECTT Treatment Group and group B the Control Group.

RETRACTED

Once a participant has been accepted into the trial, the researcher will create a photograph of the selected but unopened envelope together with the paper list of participants that does not have the new participant’s name on it. The researcher will then open the envelope and add the participant to the list and make another photograph of the list. This system of photographs is used to avoid a phenomenon in which the clinician wishes to assign participants to a particular treatment and opens more than one envelope before assigning a participant to ensure that the participant ends up in the clinician’s preferred treatment group for this participant.

### Blinding

The physical setup of the trial does not allow blinding of the practitioner or the patient. The final assessment a week after the last treatment, and the follow-up assessments, will be done by a person blinded to group allocation and treatment. The statistician performing the statistical analyses will also be blinded to group allocation and treatment.

### Interventions

The Control Group will receive the conventional doctor-directed treatment, which in this design is standard physiotherapy consisting of four weekly 50-minute sessions that use some combination of deep tissue massage, a TENS machine, electro-acupuncture, a vibrating handheld massage tool and a heat lamp Additional file 2. The control treatment will be provided by physiotherapeutic nurses. None of these treatments are recommended for CLBP [65], partly because, except for radiofrequency denervation, no intervention is recommended for CLBP [65], although massage is recommended for acute LBP and acupuncture/TENS is a popular treatment with 3000 studies of the technique [101]. There are no personnel available who are qualified in both ECTT and physiotherapy, hence the intervention and control treatments are provided by different practitioners. There is a potential confounding effect in having different practitioners but this setup avoids the possibility that the practitioners may have a bias towards either technique and would treat accordingly.

The ECTT treatment will follow the techniques provided in the ECTT training manuals [102, 103] as described earlier under Background/ECTT description.

RETRACTED

### Procedures

The hospital will contact its CLBP patients and advertise in a local newspaper and by SMS that foreign practitioners are available to offer back pain treatments. This is a normal occurrence; for example, surgeons from the US perform free cleft palate and cleft lip operations once or twice a year at the hospitals participating in the study. Additional participants are expected through word of mouth from patients who previously received ECTT and from the examination and emergency ward of the participating hospitals.

The recruited patients will be referred to the Rehabilitation, Physiotherapy and Natural Medicine Science ward, where both groups will receive their treatments.

A medical doctor at the ward will collect data on the patient’s age, gender, height, weight, level of education, chronicity (duration of chronic pain) assessment, whether they have been off work for more than 1 month, other pain sites and the inclusion and exclusion criteria, which include their current level of LBP on the VAS. If the patients are eligible to be part of the trial, they will be given the patient information and consent form to read and, if they approve, to sign.

As a next step, the patients will be assigned randomly to the Treatment or Control Groups and asked to complete the SF-36 and the Quebec scale. Each participant will then receive four weekly sessions of ECTT or the standard physiotherapy treatment. At the beginning of each treatment, each patient will be asked by an administering nurse to indicate their pain levels on the VAS. One week after the fourth and last session, all patients will be contacted by a nurse who is unaware of their group assignment. The nurse will record their pain level and give the patients the SF-36 and the Quebec scale to complete.

The treatments will take place in a large room with nurses and three translators present. The practitioners have also learnt some Vietnamese so that they can give some feedback to the participants if needed; for all other communication, a translator will be used.

The next time the ECTT practitioners visit, either in March or July, the first follow-up survey will be done. At the second visit, the second follow-up survey will be administered. The participants will receive no treatment as part of this trial during the follow-up visits.

The following treatment protocol will apply to the control group and will be administered by Vietnamese physiotherapy-trained nurses:

- Massage for 15 minutes.
- TENS machine for 15 minutes.
- Electro-acupuncture with UV heat lamp for 20 minutes.
- The TENS machine, the electro-acupuncture and the heat lamp are set at the highest level the patient is comfortable with.

RETRACTED

### Outcome measures

Outcome measures have been selected based on those chosen for previous trials of interventions on LBP [24, 104–107].

### Primary outcome measures

The primary outcome will be change in pain levels from baseline to the last treatment, and at follow-ups after 4 or 8 months and after 12 months (two follow-ups). “Pain” is defined as overall average LBP in the past week, as assessed by the VAS [87–89].

### Secondary outcome measures

Change in pain functionality after the last treatment and at follow-ups after 4 or 8 months and after 12 months will be assessed by the Quebec scale. Change in general physical and mental well-being will be measured by the SF-36 Physical Component Summary and the SF-36 Mental Component Summary [108]. The association between initial pain levels and primary and secondary outcome measures will also be investigated.

### Sample size

In the unpublished previous ECTT study, average improvements for participants with a starting pain level of at least 30 mm out of 100 mm were 28 mm, with a 20-mm standard deviation. Assuming a 15-mm improvement in the Control Group with the same standard deviation, a power (β) of 0.8 and α = 0.05, we need a sample size of 2 × 39 = 78 in total for the *t* test to have a statistically significant (*p* < 0.05) result, ignoring crossovers and withdrawals. Looking further afield at other RCTs on CLBP [104, 106, 107, 109–111], baseline standard deviations (SDs) ranged from 12 to 21 mm and post-treatment SDs ranged from 19 to 26 mm. Differences in post-treatment mean scores ranged from 2 to 25 mm. Hence, assuming a 15-mm difference is ambitious but may be realisable.

A recent review of studies on LBP [53] defined acceptable cut-off values for attrition of 20% in the short term (3 months or less) and 30% in the long term (9 months or more). Similarly, a meta-analysis by Ibrahim et al. of surgical treatment for CLBP [112] considered 20% attrition in less than 3 months acceptable. The Cochrane handbook [113] does not offer numerical guidelines. Hence, 50 participants in each group was identified as a sufficient sample size to allow for attrition of up to 20%.

Protocol violations, for example withdrawals and crossovers (from Treatment Group to Control Group or vice versa), will be managed on an intention-to-treat basis. Withdrawals may lead to missing data; however, we will endeavour to obtain follow-up data on all randomised patients, including those who withdraw. All protocol deviations and exclusions, including their reasons, will be reported for each arm of the trial.

RETRACTED

### Unadjusted and adjusted analyses

For each outcome variable, the unadjusted analysis will be designated as the primary analysis; the covariate-adjusted analysis will be designated as the secondary analysis. Adjusted analyses will incorporate the following covariates: age, sex, initial pain level, initial physical and mental health according to SF-36 scores and Quebec scores.

### Missing data

Every effort will be made to obtain data, irrespective of whether the patient completed the treatment. The analyses will be based on available data only, because mixed modelling of longitudinal data is robust to the “missing at random” missing data mechanism [114], hence meaningful results can be ascertained even when there are missing data and no substitution mechanism for missing data is needed. However, if the amount of missing data is substantial (>10%), we will investigate mechanisms of possible non-randomness of missing data.

### Statistical analysis

For each group, summary statistics will include age, gender, BMI, duration of chronic pain and status of being off work for more than 1 month, initial and ending pain levels, main SF-36 scores and Quebec scores.

The software used will be Stata version 14 or later (StataCorp, College Station, TX, USA). If the data fulfil the normalcy requirements, a simple regression analysis will be used for the Quebec and SF-36 data.

Because the pain score is longitudinal, and changes in pain levels may differ between weeks, the data analysis will use either GEE (generalized estimating equations), with time as a categorical variable, or multi-level modelling:

$$ \begin{array}{l}\mathtt{xtset}\ \mathtt{i}\mathtt{d}\ \mathtt{week}\\ {}\mathtt{xtgee}\ \mathtt{PainW}\ \mathtt{i}.\mathtt{Control}\#\#\mathtt{i}.\mathtt{week},\ \mathtt{i}\left(\mathtt{id}\right)\ \mathtt{corr}\left(\mathtt{sta}\ \mathtt{4}\right)\ \mathtt{robust}\end{array} $$

or, alternatively mixed modelling:

$$ \mathtt{mixed}\ \mathtt{PainW}\ \mathtt{i}.\mathtt{week}\#\#\mathtt{i}.\mathtt{Treatment}\ \left|\ \right|\ \mathtt{i}\mathtt{d}:,\ \mathtt{residual}\left(\mathtt{ar}\mathtt{1},\ \mathtt{t}\left(\mathtt{week}\right)\right),\ \mathtt{stddev}\ \mathtt{nolog}\ \mathtt{reml} $$

Because we are only comparing population means and not making individual predictions, the simpler GEE approach may be the more suitable.

## Discussion

### Benefits and disadvantages of the randomised controlled trial

As already described, a single phase I/phase II trial established that the ECTT intervention is safe and may be effective for chronic pain, including CLBP. Therefore, a randomised controlled trial of ECTT is warranted. The trial is to be conducted in Vietnam because two ECTT practitioners have already established a 4-year voluntary relationship, treating altogether several hundred patients twice a year in two hospitals. These two hospitals are providing the medical and logistical support for the trial and free physiotherapy sessions for the Control Group.

RETRACTED

Because of the lack of high-quality evidence for the efficacy of ECTT, at this stage it is not possible to conduct such a trial at a hospital in Australia, although this would have been the preferred option. The practitioners only have limited Vietnamese language proficiency, which reduces the possibilities for verbal communication with the participants; hence, the placebo effect from the ECTT practitioners is expected to be lower than that from the physiotherapy nurses who are administering the standard treatment and who are all Vietnamese. This may therefore lead to an understating of the effect of ECTT compared with the standard treatment.

As has been noted by experts on the conduct of business in Vietnam, “Compared to other Asian countries, Vietnamese are proud people and treating them with respect and courtesy will go a long way” [115]. Hence, a placebo effect through some patients showing extra respect to the western practitioners purely because they are westerners could well be balanced by others showing less respect, for example any war veterans among the patients, which may explain why the nationality or race of a practitioner is usually not recorded in a clinical trial.

Because only Vietnamese participants will be treated, there may be limitations in applying the results to patients from other nations. Only the SF-36 has been culturally validated for Vietnamese speakers, albeit for Vietnamese speakers who reside outside Vietnam [116]. The Quebec scale has not been culturally validated, but its simplicity may make this less of an issue.

There are no objective measures for pain, hence there is no known objective way to measure the treatment effect of an intervention on chronic non-specific LBP. All tests assess some aspect of the patient’s pain: tolerance (bending and lifting of limbs), experience (VAS), day-to-day functionality (Quebec scale, SF-36) or mental well-being (SF-36). Tests that rely on some level of participants’ pain tolerance have, as in other randomised controlled trials on LBP, not been included because they pose a danger of aggravating the participants’ condition [24, 104–107].

This study uses a randomised controlled trial design to consider whether ECTT is more effective than a standard physiotherapeutic treatment for reducing CLBP, pain functionality and mental well-being.

The study design has some limitations. First, blinding of patients and practitioners is not possible; second, the research is to be conducted in just two hospitals in Vietnam. Nevertheless, the design also has important strengths: reproducibility, the blinding of the assessor and data analyst and the incorporation of current clinical practice as a comparator. The outcome will provide evidence-based conclusions regarding the effectiveness of this low-intervention treatment for the management of patients with CLBP.

RETRACTED

## Trial status

The study is not yet recruiting as of the date of the publication.

## Additional files

Additional file 1: is the SPIRIT checklist. (DOC 123 kb)

Additional file 2: is the Template for Intervention Description and Replication (TIDieR) table. (PDF 357 kb)

## Abbreviations

BMI: Body mass index
CAM: Complementary and alternative medicine
CLBP: Chronic low back pain (low back pain for at least half of the last 180 days)
ECTT: Esoteric Connective Tissue Therapy
LBP: Low back pain
SF-36: Short Form 36

## References

[1] Hoy D, March L, Brooks P, Blyth F, Woolf A, Bain C, Williams G, Smith E, Vos T, Barendregt J (2014). The global burden of low back pain: estimates from the Global Burden of Disease 2010 study. Ann Rheum Dis.

[2] Driscoll T, Jacklyn G, Orchard J, Passmore E, Vos T, Freedman G, Lim S, Punnett L (2014). The global burden of occupationally related low back pain: estimates from the Global Burden of Disease 2010 study. Ann Rheum Dis.

[3] Hoa TTM, Darmawan J, Le Chen S, Van Hung N, Nhi CT, An TN, Damarwan J, Le CS (2003). Prevalence of the rheumatic diseases in urban Vietnam: a WHO-ILAR COPCORD study. J Rheumatol.

[4] Freburger JK, Holmes GM, Agans RP, Jackman AM, Darter JD, Wallace AS, Castel LD, Kalsbeek WD, Carey TS (2009). The rising prevalence of chronic low back pain. Arch Intern Med.

[5] Walker BF, Muller R, Grant WD (2004). Low back pain in Australian adults. Prevalence and associated disability. J Manip Physiol Ther.

[6] Health-care expenditure on arthritis and other musculoskeletal conditions 2008–09. 2014. http://www.aihw.gov.au/WorkArea/DownloadAsset.aspx?id=60129548474. Accessed 28 May 2017.

[7] Ivanova JI, Birnbaum HG, Schiller M, Kantor E, Johnstone BM, Swindle RW (2011). Real-world practice patterns, health-care utilization, and costs in patients with low back pain: the long road to guideline-concordant care. Spine J.

[8] Maniadakis N, Gray A (2000). The economic burden of back pain in the UK. Pain.

[9] Waddell G. The back pain revolution. Elsevier Health Sciences; 2004. p. 122.1st March 2004.

[10] Costa LCM, Maher CG, McAuley JH, Hancock MJ, Herbert RD, Refshauge KM, Henschke N (2009). Prognosis for patients with chronic low back pain: inception cohort study. BMJ..

RETRACTED

[11] Carey TS, Garrett JM, Jackman AM (2000). Beyond the good prognosis: examination of an inception cohort of patients with chronic low back pain. Spine.

[12] Korff MV, Deyo RA, Cherkin D, Barlow W (1993). Back pain in primary care: outcomes at 1 year. Spine.

[13] Dunn KM, Croft PR (2006). The importance of symptom duration in determining prognosis. Pain.

[14] Jones GT, Johnson RE, Wiles NJ, Chaddock C, Potter RG, Roberts C, Symmons DP, Macfarlane GJ (2006). Predicting persistent disabling low back pain in general practice: a prospective cohort study. Br J Gen Pract.

[15] Croft PR, Macfarlane GJ, Papageorgiou AC, Thomas E, Silman AJ (1998). Outcome of low back pain in general practice: a prospective study. BMJ.

[16] Nyiendo J, Haas M, Goldberg B, Sexton G (2001). Pain, disability, and satisfation outcomes and predictors of outcomes: a practice-based study of chronic low back pain patients attending primary care and chiropractic physicians. J Manip Physiol Ther.

[17] Reme SE, Hagen EM, Eriksen HR (2009). Expectations, perceptions, and physiotherapy predict prolonged sick leave in subacute low back pain. BMC Musculoskelet Disord..

[18] Airaksinen O, Brox J, Cedraschi C, Hildebrandt J, Klaber-Moffett J, Kovacs F, Mannion A, Reis S, Staal J, Ursin H (2006). Chapter 4 European guidelines for the management of chronic nonspecific low back pain. Eur Spine J..

[19] Bogduk N (2004). Management of chronic low back pain. Med J Australia.

[20] Bronfort G, Haas M, Evans R, Kawchuk G, Dagenais S (2008). Evidence-informed management of chronic low back pain with spinal manipulation and mobilization. Spine J.

[21] Bronfort G, Haas M, Evans RL, Bouter LM (2004). Efficacy of spinal manipulation and mobilization for low back pain and neck pain: a systematic review and best evidence synthesis. Spine J.

[22] Brox JI, Storheim K, Grotle M, Tveito TH, Indahl A, Eriksen HR (2008). Systematic review of back schools, brief education, and fear-avoidance training for chronic low back pain. Spine J.

[23] Cherkin DC, Sherman KJ, Deyo RA, Shekelle PG (2003). A review of the evidence for the effectiveness, safety, and cost of acupuncture, massage therapy, and spinal manipulation for back pain. Ann Intern Med.

[24] Chou R, Huffman LH (2007). Nonpharmacologic therapies for acute and chronic low back pain: A review of the evidence for an American Pain Society/American College of Physicians clinical practice guideline. Ann Intern Med.

[25] Chou R, Loeser JD, Owens DK, Rosenquist RW, Atlas SJ, Baisden J, Carragee EJ, Grabois M, Murphy DR, Resnick DK (2009). Interventional therapies, surgery, and interdisciplinary rehabilitation for low back pain: an evidence-based clinical practice guideline from the American Pain Society. Spine.

RETRACTED

[26] Chou R, Qaseem A, Snow V, Casey D, Cross JT, Shekelle P, Owens DK (2007). Diagnosis and treatment of low back pain: a joint clinical practice guideline from the American College of Physicians and the American Pain Society. Ann Intern Med.

[27] Cramer H, Haller H, Lauche R, Dobos G (2012). Mindfulness-based stress reduction for low back pain. A systematic review. BMC Complement Altern Med..

[28] Cramer H, Lauche R, Haller H, Dobos G (2013). A systematic review and meta-analysis of yoga for low back pain. Clin J Pain.

[29] Ernst E, Canter PH (2006). A systematic review of systematic reviews of spinal manipulation. J R Soc Med.

[30] Ernst E, Harkness E (2001). Spinal manipulation: a systematic review of sham-controlled, double-blind, randomized clinical trials. J Pain Symptom Manage.

[31] Ferreira ML, Ferreira PH, Latimer J, Herbert R, Maher CG (2002). Does spinal manipulative therapy help people with chronic low back pain?. Aust J Physiother.

[32] Fersum KV, Dankaerts W, O'Sullivan PB, Maes J, Skouen JS, Bjordal JM, Kvåle A (2010). Integration of subclassification strategies in randomised controlled clinical trials evaluating manual therapy treatment and exercise therapy for non-specific chronic low back pain: a systematic review. Br J Sports Med.

[33] Franke H, Franke JD, Fryer G (2014). Osteopathic manipulative treatment for nonspecific low back pain: a systematic review and meta-analysis. BMC Musculoskelet Disord..

[34] Furlan AD, Imamura M, Dryden T, Irvin E (2009). Massage for low back pain: an updated systematic review within the framework of the Cochrane back review group. Spine.

[35] Furlan AD, van Tulder M, Cherkin D, Tsukayama H, Lao L, Koes B, Berman B (2005). Acupuncture and dry-needling for low back pain: an updated systematic review within the framework of the cochrane collaboration. Spine.

[36] Furlan AD, Yazdi F, Tsertsvadze A, Gross A, Van Tulder M, Santaguida L, Gagnier J, Ammendolia C, Dryden T, Doucette S (2012). A systematic review and meta-analysis of efficacy, cost-effectiveness, and safety of selected complementary and alternative medicine for neck and low-back pain. Evid-Based Compl Alt..

[37] Guzmán J, Esmail R, Karjalainen K, Malmivaara A, Irvin E, Bombardier C (2001). Multidisciplinary rehabilitation for chronic low back pain: systematic review. BMJ.

[38] Hayden JA, van Tulder MW, Tomlinson G (2005). Systematic review: Strategies for using exercise therapy to improve outcomes in chronic low back pain. Ann Intern Med.

[39] Henchoz Y, Kai-Lik SA (2008). Exercise and nonspecific low back pain: a literature review. Joint Bone Spine.

RETRACTED

[40] Heymans MW, van Tulder MW, Esmail R, Bombardier C, Koes BW (2005). Back schools for nonspecific low back pain: a systematic review within the framework of the Cochrane collaboration back review group. Spine.

[41] Hoffman BM, Papas RK, Chatkoff DK, Kerns RD (2007). Meta-analysis of psychological interventions for chronic low back pain. Health Psychol.

[42] Hutchinson AJ, Ball S, Andrews JC, Jones GG (2012). The effectiveness of acupuncture in treating chronic non-specific low back pain: a systematic review of the literature. J Orthop Surg Res..

[43] Kamper SJ, Apeldoorn AT, Chiarotto A, Smeets RJ, Ostelo RW, Guzman J, van Tulder MW (2015). Multidisciplinary biopsychosocial rehabilitation for chronic low back pain: Cochrane systematic review and meta-analysis. BMJ..

[44] Koes BW, Assendelft WJJ, Van der Heijden GJMG, Bouter LM (1996). Spinal manipulation for low back pain: an updated systematic review of randomized clinical trials. Spine.

[45] Liddle SD, Baxter GD, Gracey JH (2004). Exercise and chronic low back pain: what works?. Pain.

[46] Macario A, Pergolizzi JV (2006). Systematic literature review of spinal decompression via motorized traction for chronic discogenic low back pain. Pain Pract.

[47] Macedo LG, Maher CG, Latimer J, McAuley JH (2008). Motor control exercise for persistent, nonspecific low back pain: a systematic review. Phys Ther..

[48] Machado LAC, de Souza MS, Ferreira PH, Ferreira ML (2006). The Mckenzie method for low back pain: a systematic review of the literature with a meta-analysis approach. Spine.

[49] Manheimer E, White A, Berman B, Forys K, Ernst E (2005). Meta-analysis: Acupuncture for low back pain. Ann Intern Med.

[50] May S, Johnson R (2008). Stabilisation exercises for low back pain: a systematic review. Physiotherapy.

[51] Orrock PJ, Myers SP (2013). Osteopathic intervention in chronic non-specific low back pain: a systematic review. BMC Musculoskelet Disord..

[52] Rainville J, Hartigan C, Martinez E, Limke J, Jouve C, Finno M (2004). Exercise as a treatment for chronic low back pain. Spine J.

[53] Rubinstein SM, van Middelkoop M, Assendelft WJJ, de Boer MR, van Tulder MW (2011). Spinal manipulative therapy for chronic low-back pain. Cochrane Database Syst Rev..

[54] Rubinstein SM, van Middelkoop M, Kuijpers T, Ostelo R, Verhagen AP, de Boer MR, Koes BW, van Tulder MW (2010). A systematic review on the effectiveness of complementary and alternative medicine for chronic non-specific low-back pain. Eur Spine J.

[55] Slade SC, Keating JL (2006). Trunk-strengthening exercises for chronic low back pain: a systematic review. J Manip Physiol Ther.

[56] Slade SC, Keating JL (2007). Unloaded movement facilitation exercise compared to no exercise or alternative therapy on outcomes for people with nonspecific chronic low back pain: a systematic review. J Manip Physiol Ther.

RETRACTED

[57] Steiger F, Wirth B, de Bruin ED, Mannion AF (2012). Is a positive clinical outcome after exercise therapy for chronic non-specific low back pain contingent upon a corresponding improvement in the targeted aspect(s) of performance? A systematic review. Eur Spine J.

[58] van Middelkoop M, Rubinstein SM, Kuijpers T, Verhagen AP, Ostelo R, Koes BW, van Tulder MW (2011). A systematic review on the effectiveness of physical and rehabilitation interventions for chronic non-specific low back pain. Eur Spine J.

[59] van Middelkoop M, Rubinstein SM, Verhagen AP, Ostelo RW, Koes BW, van Tulder MW (2010). Exercise therapy for chronic nonspecific low-back pain. Best Pract Res Clin Rheumatol.

[60] van Tulder M, Malmivaara A, Esmail R, Koes B (2000). Exercise therapy for low back pain: a systematic review within the framework of the Cochrane collaboration back review group. Spine.

[61] van Tulder MW, Cherkin DC, Berman B, Lao L, Koes BW (1999). The effectiveness of acupuncture in the management of acute and chronic low back pain: a systematic review within the framework of the Cochrane collaboration back review group. Spine.

[62] van Tulder MW, Koes B, Malmivaara A (2006). Outcome of non-invasive treatment modalities on back pain: an evidence-based review. Eur Spine J.

[63] van Tulder MW, Koes BW, Bouter LM (1997). Conservative treatment of acute and chronic nonspecific low back pain: a systematic review of randomized controlled trials of the most common interventions. Spine.

[64] Waller B, Lambeck J, Daly D (2009). Therapeutic aquatic exercise in the treatment of low back pain: a systematic review. Clin Rehabil.

[65] Low back pain and sciatica in over 16 s: assessment and management. 2016. https://www.nice.org.uk/guidance/ng59/resources/low-back-pain-and-sciatica-in-over-16s-assessment-and-management-1837521693637. Accessed 17 Apr 2017.

[66] Qaseem A, Wilt TJ, McLean RM, Forciea M, for the Clinical Guidelines Committee of the American College of Physicians. Noninvasive treatments for acute, subacute, and chronic low back pain: A clinical practice guideline from the american college of physicians. Ann Intern Med. 2017;166(7):514–30.10.7326/M16-236728192789

[67] Haldeman S, Dagenais S (2008). What have we learned about the evidence-informed management of chronic low back pain?. Spine J.

[68] Bernstein IA, Malik Q, Carville S, Ward S. Low back pain and sciatica: summary of NICE guidance. BMJ. 2017;356:i6748.10.1136/bmj.i674828062522

[69] Walker BF, Muller R, Grant WD. Low back pain in Australian adults: the economic burden. Asia Pac J Public Health. 2003;15(2):79–87. http://journals.sagepub.com/home/aph.10.1177/10105395030150020215038680

RETRACTED

[70] Buchbinder R, Blyth FM, March LM, Brooks P, Woolf AD, Hoy DG (2013). Placing the global burden of low back pain in context. Best Pract Res Clin Rheumatol.

[71] Ioannidis JP (2005). Why most published research findings are false. PLoS Med.

[72] Harris P, Rees R (2000). The prevalence of complementary and alternative medicine use among the general population: a systematic review of the literature. Complementary Ther Med.

[73] Eisenberg DM, Davis RB, Ettner SL (1998). Trends in alternative medicine use in the United States, 1990-1997: results of a follow-up national survey. JAMA.

[74] Barnes PM, Bloom B, Nahin RL. Complementary and alternative medicine use among adults and children: United States, 2007. Hyattsville, MD: US Department of Health and Human Services, Centers for Disease Control and Prevention, National Center for Health Statistics; 2008

[75] Hedley G (2008). Demonstration of the integrity of human superficial fascia as an autonomous organ. J Bodyw Mov Ther.

[76] Victoria A, Stahl JSG, Richard NT (2008). A Biomechanical analysis of the crural fascia in the feline hindlimb during locomotion and intra-muscular stimulation. J Bodyw Mov Ther.

[77] Guimberteau JC, Sentucq-Rigall J, Panconi B, Boileau R, Mouton P, Bakhach J (2005). Introduction to the knowledge of subcutaneous sliding system in humans. Ann Chir Plast Esthet.

[78] Esoteric Connective Tissue Therapy. 2016. https://www.universalmedicine.com.au/services/healing-therapies/connective-tissue-therapy. Accessed 17 Jul 2016.

[79] Esoteric Connective Tissue Therapy. 2016. http://www.esotericwomenshealth.com/esoteric-connective-tissue-therapy.html. Accessed 17 Jul 2016.

[80] Esoteric Connective Tissue Therapy. 2016. http://web.archive.org/web/20170216120951/. http://medicinalhealing.com.au/services/esoteric-connective-tissue-therapy. Accessed 17 Jul 2016.

[81] Physical pain and the miracle of Esoteric Connective Tissue Therapy. 2014. https://truthaboutuniversalmedicine.com/2014/06/22/physical-pain-and-the-miracle-of-esoteric-connective-tissue-therapy/. Accessed 17 Jul 2016.

[82] What students say about connective tissue therapy. 2016. http://www.universalmedicine.net/about-connective-tissue-therapy.html. Accessed 17 Jul 2016.

[83] Langevin HM, Stevens-Tuttle D, Fox JR, Badger GJ, Bouffard NA, Krag MH, Wu J, Henry SM (2009). Ultrasound evidence of altered lumbar connective tissue structure in human subjects with chronic low back pain. BMC Musculoskelet Disord.

[84] Oschman JL. Energy medicine in therapeutics and human performance. Elsevier Science. Published online 17 June 2003.

RETRACTED

[85] Code of Ethics and Conduct. 2009. http://esoteric-healing.com/system/files/EPA-information-pack/PDFs/EPA-Code-of-Ethics.pdf. Accessed 1 Aug 2016.

[86] Code of Ethics and Conduct 4th edition. 2014. http://web.archive.org/web/20160421032807/http://www.catholiccare.org/sites/default/files/Code%20of%20Ethics%20and%20Conduct.pdf. Accessed 23 Jul 2016.

[87] Hawker GA, Mian S, Kendzerska T, French M (2011). Measures of adult pain. Arthr Rheum-Arthr.

[88] Price DD, McGrath PA, Rafii A, Buckingham B (1983). The validation of visual analogue scales as ratio scale measures for chronic and experimental pain. Pain.

[89] Collins SL, Moore RA, McQuay HJ (1997). The visual analogue pain intensity scale: what is moderate pain in millimetres?. Pain.

[90] Deyo RA, Dworkin SF, Amtmann D, Andersson G, Borenstein D, Carragee E, Carrino J, Chou R, Cook K, DeLitto A (2014). Report of the NIH Task Force on research standards for chronic low back pain. Spine J.

[91] National Statement on Ethical Conduct in Human Research 2007 (Updated May 2015). 2015. http://www.nhmrc.gov.au/_files_nhmrc/publications/attachments/e72_national_statement_may_2015_150514_a.pdf. Accessed15 Jul 2016.

[92] Kopec JA, Esdaile JM, Abrahamowicz M, Abenhaim L, Wood-Dauphinee S, Lamping DL, Williams JI (1995). The Quebec Back Pain Disability Scale: measurement properties. Spine.

[93] Kopec JA, Esdaile JM, Abrahamowicz M, Abenhaim L, Wood-Dauphinee S, Lamping DL, Williams JI (1996). The Quebec Back Pain Disability Scale: conceptualization and development. J Clin Epidemiol.

[94] Kelly A-M (2001). The minimum clinically significant difference in visual analogue scale pain score does not differ with severity of pain. Emerg Med J.

[95] Bennell KL, Egerton T, Pua Y-H, Abbott JH, Sims K, Metcalf B, McManus F, Wrigley TV, Forbes A, Harris A (2010). Efficacy of a multimodal physiotherapy treatment program for hip osteoarthritis: a randomised placebo-controlled trial protocol. BMC Musculoskelet Disord.

[96] Ostelo RWJG, Deyo RA, Stratford P, Waddell G, Croft P, Von Korff M, Bouter LM, de Vet HC (2008). Interpreting change scores for pain and functional status in low back pain: towards international consensus regarding minimal important change. Spine.

[97] Ware JE, Kosinski M, Dewey JE, Gandek B. SF-36 Health Survey: Manual and interpretation guide (Book) Quality Metric Inc., Lincoln RI USA; 2000.

[98] Angst F, Aeschlimann A, Stucki G (2001). Smallest detectable and minimal clinically important differences of rehabilitation intervention with their implications for required sample sizes using WOMAC and SF-36 quality of life measurement instruments in patients with osteoarthritis of the lower extremities. Arthrit Rheum-Arthr.

RETRACTED

[99] Hoy D, Brooks P, Blyth F, Buchbinder R (2010). The epidemiology of low back pain. Best Pract Res Clin Rheumatol.

[100] Create a blocked randomisation list. 2016. https://www.sealedenvelope.com/simple-randomiser/v1/lists. Accessed 28 May 2017.

[101] Colquhoun D, Novella SP. Acupuncture is theatrical placebo. Anesthesia & Analgesia. 2013;116(6):1360-3.10.1213/ANE.0b013e31828f2d5e23709076

[102] Benhayon S, Benhayon C. Esoteric Connective Tissue Therapy advanced level 2; 2014. Instruction manual, paper only. Serge Benhayon; 2000.

[103] Benhayon S, Benhayon C. Esoteric Connective Tissue Therapy advanced level 1; 2014. Instruction manual, paper only. Serge Benhayon; 2000.

[104] Brox JI, Sørensen R, Friis A, Nygaard Ø, Indahl A, Keller A, Ingebrigtsen T, Eriksen HR, Holm I, Koller AK (2003). Randomized clinical trial of lumbar instrumented fusion and cognitive intervention and exercises in patients with chronic low back pain and disc degeneration. Spine.

[105] Cherkin DC, Sherman KJ, Kahn J, Wellman R, Cook AJ, Johnson E, Erro J, Delaney K, Deyo RA (2011). A comparison of the effects of 2 types of massage and usual care on chronic low back pain: a randomized, controlled trial. Ann Intern Med.

[106] Ferreira ML, Ferreira PH, Latimer J, Herbert RD, Hodges PW, Jennings MD, Maher CG, Refshauge KM (2007). Comparison of general exercise, motor control exercise and spinal manipulative therapy for chronic low back pain: a randomized trial. Pain.

[107] Fritzell P, Hägg O, Wessberg P, Nordwall A, Swedish Lumbar Spine Study G (2001). 2001 Volvo Award Winner in Clinical Studies: Lumbar fusion versus nonsurgical treatment for chronic low back pain: a multicenter randomized controlled trial from the Swedish Lumbar Spine Study Group. Spine.

[108] McHorney CA, Ware Jr JE, Raczek AE. The MOS 36-Item Short-Form Health Survey (SF-36): II. Psychometric and clinical tests of validity in measuring physical and mental health constructs. Med Care. 1993;31(3):247–63.10.1097/00005650-199303000-000068450681

[109] Haake M, Müller H-H, Schade-Brittinger C, Basler HD, Schäfer H, Maier C, Endres HG, Trampisch HJ, Molsberger A (2007). German Acupuncture Trials (GERAC) for chronic low back pain: randomized, multicenter, blinded, parallel-group trial with 3 groups. Arch Intern Med.

[110] Majchrzycki M, Kocur P, Kotwicki T (2014). Deep tissue massage and nonsteroidal anti-inflammatory drugs for low back pain: a prospective randomized trial. ScientificWorldJournal..

[111] van Kleef M, Barendse GA, Kessels A, Voets HM, Weber WE, de Lange S (1999). Randomized trial of radiofrequency lumbar facet denervation for chronic low back pain. Spine.

RETRACTED

[112] Ibrahim T, Tleyjeh IM, Gabbar O (2008). Surgical versus non-surgical treatment of chronic low back pain: a meta-analysis of randomised trials. Int Orthop.

[113] Green S. Cochrane handbook for systematic reviews of interventions version 5.1. 0. The Cochrane Collaboration. 2011. http://training.cochrane.org/handbook. Accessed 15 Jul 2016.

[114] Verbeke G, Molenberghs G. Linear mixed models for longitudinal data. Springer Science & Business Media; 2009. p. 285.

[115] Meyer KE, Tran YTT, Nguyen HV. Doing business in … Vietnam. Thunderbird International Business Review. 2006;48(2):263–90.

[116] Watkins RE, Plant AJ, Sang D, O'Rourke T, Gushulak B. Development of a Vietnamese version of the Short Form-36 Health Survey. Asia Pac J Public Health. 2000;12(2):118–23. http://journals.sagepub.com/home/aph.10.1177/10105395000120021111841039

[117] Hrynaszkiewicz I, Norton ML, Vickers AJ, Altman DG (2010). Preparing raw clinical data for publication: guidance for journal editors, authors, and peer reviewers. Trials.

